# Context-Fused Guidance for Image Captioning Using Sequence-Level Training

**DOI:** 10.1155/2022/9743123

**Published:** 2022-01-05

**Authors:** Junlong Feng, Jianping Zhao

**Affiliations:** School of Computer Science and Technology, Changchun University of Science and Technology, Changchun, China

## Abstract

Recent image captioning models based on the encoder-decoder framework have achieved remarkable success in humanlike sentence generation. However, an explicit separation between encoder and decoder brings out a disconnection between the image and sentence. It usually leads to a rough image description: the generated caption only contains main instances but neglects additional objects and scenes unexpectedly, which reduces the caption consistency of the image. To address this issue, we proposed an image captioning system within context-fused guidance in this paper. It incorporates regional and global image representation as the compositional visual features to learn the objects and attributes in images. To integrate image-level semantic information, the visual concept is employed. To avoid misleading decoding, a context fusion gate is introduced to calculate the textual context by selectively aggregating the information of visual concept and word embedding. Subsequently, the context-fused image guidance is formulated based on the compositional visual features and textual context. It provides the decoder with informative semantic knowledge. Finally, a captioner with a two-layer LSTM architecture is constructed to generate captions. Moreover, to overcome the exposure bias, we train the proposed model through sequence decision-making. The experiments conducted on the MS COCO dataset show the outstanding performance of our work. The linguistic analysis demonstrates that our model improves the caption consistency of the image.

## 1. Introduction

Image captioning, which analyses and converts the image content into a natural language description automatically, is drawing considerable attention in the artificial intelligence field. As a typical multimodal task, the image captioning system combines both computer vision and natural language processing. Therefore, it should not only recognize the salient image objects and other visual properties (attributes, locations, and relations) but also depict the image content with natural and coherent descriptions [1]. Over the past few years, image captioning task has been applied on a wide area of aspects, such as assistance for visually impaired people [2].

For current image captioning system, the encoder-decoder architecture has been a widely adopted pipeline for its conspicuous performance. In general, it employs a convolutional neural network (CNN) to encode the image into a set of feature vectors and a long short-term memory (LSTM) network to generate the captions. Moreover, to steer the model into focusing and capturing informative visual features on a particular image region, the attention mechanisms are introduced as well [3–5].

The encoder-to-decoder framework has achieved remarkable advances in humanlike caption generating, but there are still some issues to be concerned.

First, to capture the visual and textual information simultaneously, some prior networks [3, 4] were designed to learn the sentence structure at a global level. Strictly, the generated caption can only depict the image roughly because during decoding, the network may discard some useful image objects or scenes unexpectedly. This reduces the consistency between image and text description. As a solution, the guidance vector is adopted [6–8]. In [6], the time-independent guidance was implemented as a joint text-image embedding. However, as pointed out in [7], their approach is short of consideration from two aspects: (1) from the view of computer vision, visual evidence is not always essential for the decoder because the description sentence usually contains salient objects that correspond to visual features; (2) the explicit separation between encoder and decoder usually leads to a representational disconnect between the learned feature vectors and generated captions. To handle these issues, they constructed a semantic image guidance, which is conditioned on textual context and image features. It provides the decoder with semantic information from *n*-gram word and sentence levels. Through this, the generated captions include richer image instances than [6]. Nevertheless, their approach neglects the information about motions and locations of image objects. In addition, although the sentence-level guidance achieved the best performance, it is not a very efficient approach because of the prepositions, articles, and conjunctions in the sentence. Considering the fact that the instances in region image are not always corresponding to the words in the vocabulary, in [8], they concatenated the global image representation with the visual concept [9] as the guidance vector. The visual concept is a set of frequent words that describe the salient image objects, which enhances the correlation between image and text at regional level. However, there is a latent drawback: an inappropriate word in visual concept will mislead the language model to generate unexpected captions.

Second, as indicated in [10], for the models trained with maximum likelihood estimation (MLE), the vanilla encoder-decoder framework may cause the problem of exposure bias. The error accumulation caused by MLE probably results in a word mismatching during caption generating. To address this issue, the reinforcement learning (RL) strategy is introduced in the image captioning task. However, due to the high variance of gradient estimation, it is extremely difficult to train the model with RL strategy directly. To meet this criterion, the self-critical sequence training (SCST) framework [11] is proposed to apply the RL strategy by sequence-level training. During the inference stage, SCST utilizes the generating samples as the baseline to normalize the rewards. Consequently, the network can use nondifferentiable sequence-level metrics (e.g., CIDEr [12]) to evaluate the language quality rather than the cross-entropy loss in word level. Based on this framework, a number of approaches were proposed [13–15]. Particularly, in [14], they proposed the CAVP to accomplish the visual decision-making task. The CAVP captures the visual context that is crucial for compositional reasoning and attends to complex visual compositions over time. Through this, it significantly boosted the caption consistency to image content.

Therefore, to boost the caption consistency of image by utilizing reasonable semantic information and informative visual features, an image captioning system within context-fused guidance (CFG) is proposed in this paper. The main idea is illustrated in Figure 1. The CFG utilizes compositional visual features for multilevel image learning.

By the context fusion gate, CFG adaptively combines the visual concept and word embedding. Using the context-fused image guidance, our model can generate captions with comprehensive descriptions. In short, the main contributions in this paper are as follows:

1. An image captioning system using sequential decision-making is proposed for a comprehensive caption generation.
2. A context-fused image guidance is formulated to improve the caption consistency of image. It selectively aggregates the semantic information from the visual concept and word embedding.
3. Evaluation on the MS COCO dataset shows that our approach outperforms most standard metrics. The linguistic analysis demonstrates that our method enhances the correlation of generated captions and images.

## 2. Related Works

### 2.1. Image Captioning

In the past few years, image captioning systems based on encoder-decoder framework have been deeply investigated [3, 16]. In [16], they employed a CNN to encode the image and a recurrent neural network to output a sequence of words. Subsequently, many works were proposed to improve and extend this framework. In [17], they proposed a recurrent fusion network (RFNet) to exploit the complementary information from multiple encoders to understand the image comprehensively. In [18], they extracted the image features at multiple levels to learn accurate subject predictions. As a very recent investigation [19], the editing network generates the image description by refining an existing caption rather than generating a new caption from scratch.

Inspired by the attention mechanism applied in machine translation, several attention-based image captioning systems were proposed. In [3], they integrated the decoder with the proposed hard and soft attention mechanism to capture the highlighting spatial image regions. In [4], they constructed a combined bottom-up and top-down attention mechanism. It calculates the attention feature vectors of the objects and other salient regions in image. In [5], the attention-on-attention module employs an attention gate to transform the result from a standard attention mechanism. Moreover, to improve the semantic representation of the generated captions, some approaches also focused on utilizing specific semantic attribute, such as the visual concept [9]. In [8], the guidance vector is equipped with the visual concept to provide the decoder with high-level semantic information. In [20], they proposed a hierarchical attention network to enhance the caption richness by incorporating the visual concept and other visual features.

### 2.2. Sequential Decision-Making

The models trained on vanilla CNN-LSTM framework often result in the problem of exposure bias [10]. To mitigate this, the reinforcement learning was applied on image captioning by introducing sequential decision-making: agent takes account of the actions, states, and rewards in further sequences. In the case of image captioning, the action corresponds to choosing the next word and image; the state can be the visual context, previous prediction, and other information. The rewards can be any evaluation metric, such as BLEU-N [21] and CIDEr [12]. Several works have applied the sequential decision-making. In [10], the REINFORCE is used to optimize a user-specified evaluation metric during training directly. However, it lacks adequate generalities to other evaluation metrics. In [11], the self-critical sequence training (SCST) framework is proposed. In SCST, the generated captions are evaluated at sentence level. Afterwards, in [13], they incorporated a discriminative loss component into the training objective to produce the caption with high discriminability. To capture crucial compositional information in image, CAVP [14] was proposed to capture complex visual compositions over time. Recently, the B-SCST [15] extended the SCST framework for image captioning models by incorporating Bayesian inference. From the distribution obtained by a Bayesian DNN model, B-SCST generates the baseline reward by averaging predictive quality metrics.

## 3. Proposed Approach

In this section, we introduce the proposed CFG network in detail. As the architecture presented in Figure 2, our model consists of five components: (1) a text encoder, which encodes the visual concept; (2) an image encoder, which encodes the region image features; (3) an attention module, which calculates the attentive compositional visual features; (4) a guidance formulation module, which obtains the fused textual context through the context gate and calculates the context-fused image guidance; and (5) a captioner, which is an extension of the top-down captioner [4] for caption generating.

### 3.1. Text Encoder

As the visual concept reveals the objects in images explicitly, we introduce it to offset the separation between image and text. In this paper, the visual concept is denoted as *A*={*a*_1_, *a*_2_,…, *a*_*m*_}, *a*_*j*_ ∈ *ℝ*^*m* ×*E*^, where *m* is the count of the words in visual concept and *E* is the dimension of word embedding. Specifically, as the word *a*_*j*_ is isolated, therefore a unidirectional LSTM is employed as the text encoder to deal with *A* as follows:

(1) $$\begin{array}{c} w=\text{LSTM}\left(E\left(A\right)\right), \end{array}$$

where *E*(·) is the word embedding layer and *w* ∈ ℝ^*m* × *H*^, where *H* is the size of hidden state. *w* indicates the encoding semantic vectors of each word in *A*. It will be used to calculate the fused textual context in the guidance formulation module.

### 3.2. Image Encoder

For the given image *I*, to learn the visual information about objects, attributes, and relations, a pretrained Faster R-CNN [22] is adopted to extract the region image representation *r* as follows:

(2) $$\begin{array}{c} r=W^{I}\left[\text{CNN}\left(I\right)\right], \end{array}$$

where  *r*={*r*_1_, *r*_2_,…, *r*_*k*_}, *r*_*i*_ ∈ ℝ^2048^, presents the semantic information of an image region and *k* indicates the number of selected ROIs according to the ranking scores. To reduce the calculate consumption, a transformation matrix *W*^*I*^ ∈ ℝ^ *H*×2048^ is applied on *r* to convert its dimension to *r* ∈*ℝ*^*k*×*H*^. Consistent with prior works, the image representation at global level is formulated by a mean-pooling operation as follows:

(3) $$\begin{array}{c} \bar{r}=\frac{1}{k}\sum_{i=1}^{k}r_{i}, \end{array}$$

where $\bar{r}\in {\mathbb{R}}^{H}$. Both *r* and $\bar{r}$ are used to compute the attentive compositional visual features.

### 3.3. Compositional Visual Features

The compositional visual features contain the image information at regional and global levels. As shown in Figure 2 (framed in blue), for the image feature vectors *r* and $\bar{r}$, an additive attention mechanism is applied to reduce the variance caused by sampling diverse image regions. Without loss of generality, we first introduce the general formulation of the attention computation used in this paper:

(4) $$\begin{array}{c} f_{\text{att}}\left(\pi ,q,h_{t}\right)=\text{softmax}\left(w_{\pi }^{T}\tanh\left(W_{q}^{\pi }q+W_{h}^{\pi }h_{t}\right)\right), \end{array}$$

where *π* indicates the attentive weight of the query vector *q*, and *h*_*t*_ stands for the hidden state output from LSTM unit. *w*_*π*_^*T*^, *W*_*q*_^*π*^, and *W*_*h*_^*π*^ are the parameters to be learned. Accordingly, for the region image feature *r*, the attention computation is presented as follows:

(5) $$\begin{array}{c} \alpha_{t}=f_{\text{att}}\left(\pi =\alpha ,q=r,h_{t}^{v}\right). \end{array}$$

Here, the parameters *w*_*α*_^*T*^ ∈ *ℝ*^*D*^, *W*_*r*_^*α*^ ∈ *ℝ*^*D*×*H*^, and *W*_*h*_^*α*^ ∈ *ℝ*^*D*×*H*^ in this case, *D* indicates the dimension of attention layer, and *h*_*t*_^*v*^ is the hidden state from attention LSTM. Then, the attentive region image feature *z*_*t*_^*r*^ is computed as follows:

(6) $$\begin{array}{c} z_{t}^{r}=\sum_{i=1}^{k+1}\alpha_{i,t}\cdot r, \end{array}$$

where *z*_*t*_^*r*^ ∈ ℝ^*H*^. Particularly, in contrast to previous works that only integrate the global image representation in the first LSTM layer, similar to equation (5), $z_{t}^{\bar{r}}$ is computed as the attentive vectors of $\bar{r}$. Then, we combine *z*_*t*_^*r*^  with $z_{t}^{\bar{r}}$ as the compositional visual features:

(7) $$\begin{array}{c} V_{\text{comp}}=\left[z_{t}^{r};z_{t}^{\bar{r}}\right], \end{array}$$

where [; ] indicates the vector concatenation. The attentive compositional visual feature *z*_*t*_^*c*^ is obtained as follows:

(8) $$\begin{array}{c} \beta_{t}=f_{\text{att}}\left(\pi =\beta ,q=V_{\text{comp}},h_{t}^{v}\right),\\ z_{t}^{c}=\sum_{i=1}^{k+1}\beta_{i,t}\cdot V_{\text{comp}}, \end{array}$$

where the trained parameters *w*_*β*_^*T*^ ∈ *ℝ*^*D*^,  *W*_*V*_^*β*^ ∈ *ℝ*^*D*×*H*^, and  *W*_*h*_^*β*^ ∈ *ℝ*^*D*×*H*^ here. In comparison to *z*_*t*_^*r*^, the decoder can capture more comprehensive visual information from *z*_*t*_^*c*^ at each decoding step. Additionally, *z*_*t*_^*c*^ is also utilized to modulate the guidance vectors.

### 3.4. Guidance Formulation

In [7], Zhou et al. conditioned the guidance information on the current word *W*_*e*_(*y*_*t*_) and used the text-conditional image feature *V* as the guidance:

(9) $$\begin{array}{c} g_{t}=\tanh\left(V⊙W_{e}\left(y_{t}\right)\right), \end{array}$$

where *W*_*e*_(·) is a text-conditional embedding matrix. Through this, the model can focus on a part of the semantic image feature when capturing a specific word. In this paper, we extend this formulation with the visual concept vector *w*. Intuitively, if modulating the semantic image guidance *g*_*t*_ on *w* only, it may mislead the generating process because of the latent inappropriate word in visual concept set. Hence, it is essential to adaptively incorporate the semantic information from word embedding and visual concept. Inspired by [23], a context fusion gate is introduced. The structure is presented in Figure 3. By this component, our model can learn how much to attend to the context from two different sources. Utilizing the word embedding and visual concept, the context fusion gate is defined as follows:

(10) $$\begin{array}{c} s_{t}=f_{t}⊙\left(W_{w}z_{t}^{w}\right)+\left(1-f_{t}\right)⊙\;\tanh\left(W_{t}\left[E\left(y_{t}\right)\right]\right), \end{array}$$

where *s*_*t*_ is the fused textual context. *W*_*w*_ ∈ ℝ^*E*×*H*^ and *W*_*t*_ ∈ ℝ^*E*×*E*^ are the weight matrix; ⊙ indicates the elementwise multiplication. The factor *f*_*t*_ ∈ (0, 1) is calculated by a sigmoid activation function *σ* as follows:

(11) $$\begin{array}{c} f_{t}=\sigma \left(W_{f}\left[z_{t}^{w};E\left(y_{t}\right)\right]\right), \end{array}$$

where *W*_*f*_ is the transformation matrix. *z*_*t*_^*w*^ indicates the attentive semantic vector, which is computed as follows:

(12) $$\begin{array}{c} \gamma_{t}=f_{att}\left(\pi =\gamma ,q=w,h_{t}^{v}\right),\\ z_{t}^{w}=\sum_{i=1}^{m+1}\gamma_{i,t}\cdot w, \end{array}$$

where the parameter *w*_*γ*_^T^ ∈ ℝ^*D*^, *W*_*w*_^*γ*^ ∈ ℝ^*D*×*H*^, and *W*_*h*_^*γ*^ ∈ ℝ^*D*×*H*^. Through this, *z*_*t*_^*w*^ is equipped with the attentive visual information. Taking *V*_comp_ and *s*_*t*_, the context-fused image guidance is formulated as follows:

(13) $$\begin{array}{c} g_{t}=\tanh\left(V_{\text{comp}}⊙W_{s}\left(s_{t}\right)\right), \end{array}$$

where *W*_*s*_ ∈ ℝ^*E*×*H*^ is a transformation matrix. In comparison to equation (9), the context-fused image guidance *g*_*t*_ contains richer visual and textual context. It will be passed into the captioner as a time-dependent variable.

### 3.5. Captioner

The captioner consists of two separated LSTM networks: attention LSTM (AttLSTM) and language LSTM (LangLSTM). The input of AttLSTM is defined as the concatenation of previous word embedding vector *E*(*y*_*t*−1_), the previous hidden state *h*_*t*−1_^*l*^ from the LangLSTM, the visual concept vector *w*, and the image representation $\bar{r}$. That is,

(14) $$\begin{array}{c} {\text{X}}_{t}=\left[h_{t-1}^{l};\bar{r};w;E\left(y_{t-1}\right)\right],\\ h_{t}^{v}=\text{AttLSTM}\left({\text{X}}_{t},h_{t-1}^{v}\right), \end{array}$$

where *h*_*t*_^*v*^ is used to attend over the visual features and semantic vectors, respectively. AttLSTM provides the LangLSTM with the feature vectors at the global level. In LangLSTM, the network focuses on generating the caption with both compositional, image feature *V*_comp_ and context-fused image guidance *g*_*t*_:

(15) $$\begin{array}{c} X_{t}^{L}=\left[V_{\text{comp}};h_{t}^{v};g_{t}\right],\\ h_{t+1}^{l}=\text{LangLSTM}\left(X_{t}^{L},h_{t}^{l}\right). \end{array}$$

Then, we apply a multilayer perceptron (MLP) following by a softmax layer on hidden state *h*_*t*_^*l*^ to obtain the probability distribution of each words as follows:

(16) $$\begin{array}{c} {\hat{y}}_{t}∼p_{t}=\text{softmax}\left(\text{MLP}\left(h_{t}^{l}\right)\right), \end{array}$$

where each value of *p*_*t*_ indicates the probability of corresponding word in vocabulary. Overall, our proposed network takes full advantage of image and text information to generate captions elaborately.

### 3.6. Training Strategy

Consistent with prior works [11], the sequence-level training strategy in this paper can be decomposed into two stages: the standard supervised learning with cross-entropy (XE) loss and the reinforcement learning with a self-critical reward. The XE loss is formulated as follows:

(17) $$\begin{array}{c} L\left(\theta \right)=-\sum_{t=1}^{N}\log\;p_{\theta }\left(y_{t}|y_{1:t-1}\right), \end{array}$$

where *N* is the length of a generated caption, *y*_1:*t*−1_ is a target ground-truth sequence, and *θ* indicates the model parameters. The supervised model is trained by minimizing this value. Then, the one with best performance is chosen as the initial network for next training stage. During reinforcement learning, the negative expected reward is minimized as follows:

(18) $$\begin{array}{c} L\left(\theta \right)=-E_{y^{s}∼p_{\theta }}\left[r\left(y_{1:T}\right)\right], \end{array}$$

where *r*(·) is the standard metric evaluation (CIDEr [12] in this paper). According to SCST [11], the gradient of *L*(*θ*) can be approximated as follows:

(19) $$\begin{array}{c} \nabla_{\theta }L\left(\theta \right)\approx -\left(r\left(y_{1:T}^{s}\right)-r\left({\hat{y}}_{1:T}\right)\right)\nabla_{\theta }\log\;p_{\theta }\left(y_{1:T}^{s}\right), \end{array}$$

where *y*_1:*T*_^*s*^ is the caption sampled from the word distribution and ${\hat{y}}_{1:T}$ is the generated caption by greedy searching. The resulting reward signal *r*(*y*_1:*T*_^*s*^)−$r\left({\hat{y}}_{1:T}\right)$ can be treated as a baseline score. The probability of each word in the sampled captions will be increased if  *r*(*y*_1:*T*_^*s*^) is higher than $r\left({\hat{y}}_{1:T}\right)$, and vice versa.

## 4. Experiments

In this section, the dataset and evaluation metrics are introduced first. Then, the implementation details and the comparing models are described. Finally, we discuss the quantitative and qualitative experiments.

### 4.1. Dataset and Metrics

The MS COCO dataset [24] is one of the most popular benchmark datasets for image captioning task. There are 82,783 images in training set, 40,504 images in validation set, and 40,775 images in test set, respectively. For a fair comparison, the dataset using “Karpathy” split (http://cs.stanford.edu/people/karpathy/deepimagesent/) is adopted in this paper. It contains 113,287 images for training, 5000 images for validation, and 5000 images for test, respectively. The statistics of these two splits are summarized in Table 1. The COCO evaluation toolkit (https://github.com/tylin/coco-caption) is used to report the captioning performance across following metrics: BLEU-N (*N* = 1, 2, 3, 4) [21], METEOR [25], ROUGHE-L [26], CIDEr [12], and SPICE [27]. In particular, SPICE is defined over the tuples divided into several categories, such as objects, relations, and attributes. It shows a reasonable correlation with human judgments. All of these metrics with a larger score indicate a better effect.

### 4.2. Implementation Details

#### 4.2.1. Preprocessing

For the region image representation, we use the bottom-up features provided by [4] which extracted top *k* = 36 features in each image as salient regions. The visual concept is detected by a pretrained model [9]. Only object attribute (nouns) is preserved. We convert all the sentences to lowercase, replace the punctuation with space, and preserve the captions with a length less than 16. The words that occurred less than five times are removed. As a result, there are 10,369 words left in the vocabulary.

#### 4.2.2. Parameter Settings

Only top five attributes in visual concept set are preserved, namely, *m* = 5. The dimension *E* of word embedding layer is set to 1000. The attention layer size *D* is set to 1024. For AttLSTM and LangLSTM, the dimension *H* of hidden state and memory cell is set to 1300. During supervised learning with XE loss, Adam optimizer [28] is adopted with the initial learning rate 5*e* − 4. We shrink it by 0.8 every 3 epochs. During reinforcement training, the Adam optimizer [28] is initialized with learning rate 5*e* − 5. We trained the network for 30 epochs with batch size 80 during the first stage. During sequence-level training, we trained the model for 50 epochs with batch size 100. If there is no improvement for 5 epochs during XE training and 8 epochs during sequence-level training, the process is stopped. The whole training takes about 30 hours on a Linux server with an NVIDIA RTX 2080Ti GPU.

#### 4.2.3. Model for Comparison

The following models are chosen for comparison: (1) NIC [16], which is a vanilla CNN-LSTM image captioning model; (2) SCST [11], which uses nondifferentiable metric for optimization; (3) up-down [4], which employs a bottom-up attention mechanism; (4) RFNet [17], which outputs the captions through multiple connections of CNN and LSTM; (5) HAN [20], which uses the hierarchy features to extend the caption richness; and (6) RAtt-Soft [29], which integrates the visual relationship attention and region features to enhance caption generating.

In particular, as the visual features in [7] are extracted by a different CNN, to investigate the performance of different guidance formulation, we also conduct a study on the following ablation models: (1) CFG_*V*_, which only preserves the compositional visual feature and removes the visual concepts, context fusion gate, and context-fused image guidance. (2) CFG_*E*_, which adopts the guidance defined in equation (9) and removes the visual concept, and context fusion gate. It is a 1-gram word-level guidance. (3) CFG_*A*_, in which the factor *f*_*t*_ is removed. The fused textual context *s*_*t*_ is computed by a vector addition directly. Their performance will be discussed in the Ablation Studies section.

### 4.3. Quantitative Analysis

The evaluation results on the test portion of the Karpathy splits are summarized in Tables 2 and 3. All the scores were inferred by beam searching with size 3. For the cross-entropy loss training (Table 2), our model achieves competitive scores with RAtt-Soft [29]. For the sequence-level optimization (Table 3), our model obtains the scores with advantages across all metrics except for ROUGE-L and SPICE. Optimized by CIDEr, the scores of CFG on all metrics are increased in Table 3. Especially the score on CIDEr is improved from 114.0 to 125.4. The comparison results indicate our model can effectively improve the captioning performance by leveraging the compositional visual feature and context-fused image guidance. Besides, by sequence-level training, our network can significantly promote the results on each evaluation metric and outperform other models. However, it also should be noted that our model fails to achieve an advantage score on SPICE metric on both Table 2 and Table 3. As mentioned, SPICE is defined over the objects, relations and attributes. In [29], RAtt-Soft utilizes the scene graph and visual relation features to precisely map visual relationship information to the semantic description. This indicated a limitation of our proposed network.

### 4.4. Qualitative Analysis

For an intuitive presentation of the image captioning effect of the model with different guidance formulation, some examples are shown in Figure 4. Compared to CFG_*E*_, the full model CFG can understand the image with detected salient objects (*with a rainbow*, *holding a racket*, *next to glass of beer*, and *with luggage*), but CFG_*E*_ neglects these instances and focuses on the main content of the images. In addition, CFG can better recognize the object *remote control*, while CFG_*E*_ mistakes it as *computer keyboard*. For the last image, CFG exactly describes the image with clear objects *pizza*, *broccoli*, and *vegetables*, while CFG_*E*_ just captures the object *broccoli* and depicts the image at a general level. These examples demonstrate that, in comparison to the guidance modulated on text-conditional embedding, the context-fused guidance is more advantageous to boost the model to depict the image comprehensively. Nevertheless, there are also several shortages in our proposed network, shown as the images presented in red frame. For the first image, our CFG succeeds in depicting the image with main instances, but it misunderstands the “desk” as “table” and generated inappropriate relation information “standing around a table.” Similarly, in the last image, our model depicts the image with an incorrect position phrase “in the water.” This indicates our network is insufficient to reason accurate relationships, especially among multiply image objects. One possible solution is to introduce the scene graph [30], which contains complex structural representation of image and sentences.

In Figure 5, we visualized the probabilities of the words the generated sentence and visual concept set, along with the object attention map, respectively. It can be found that the visual concepts are well applied to generate the captions. In the first example, the salient instances (*man*, *horse*, *filed*, and *cows*) are captured and the predicted words are highly corresponding to the detected visual concepts with high probabilities. The image content is well depicted by the generated sentence. This indicates that our model can exploit the high-probability visual concept to generate the relevant words in captions. For the second image, the weights of “bike” (0.34) and “sunset” (0.33) are much lower those of “man” (0.86) and “dock” (0.93), but our model can also reason them as the appropriate words in the caption, which enhances the comprehensiveness of text description. This shows the advantage of the context fusion gate. By selectively fusing the information of the visual concept and word embedding, it can address the issue of misleading decoding as much as possible. Moreover, both these samples demonstrate that our model is able to keep a better consistency with the image content.

### 4.5. Ablation Studies

The evaluation results of the ablations are given in Table 4. Compared to CFG_*V*_, CFG_*E*_ boosts the SPICE from 20.3 to 20.5 on cross-entropy training category, respectively. It suggests the effect of the text-conditional guidance to improve image captioning. In comparison to CFG_*E*_, CFG_*A*_ achieved weak advantage results on cross-entropy training. After CIDEr optimization, the scores of BLEU4 and SPICE are boosted from 37.8 to 38.1 and 21.1 to 21.4, respectively. Among these models, CFG still achieved the best performance across all metrics. Particularly, the CDIEr score was significantly improved after sequence-level training. These indicate the following: (1) the introduced visual concept is helpful to boost image captioning. (2) The compositional visual feature and fused textual context are effective to improve the captioning quality. (3) The context fusion gate is beneficial to integrate the context from different sources for a better image captioning performance.

## 5. Conclusions

In this paper, an image captioning system within fused context guidance is proposed to enhance caption consistency of image. By the compositional visual feature, context fusion gate, and context-fused image guidance, our model further boosts the caption consistency of image. Extensive experiments demonstrate that our proposed model significantly improves the baseline method and outperforms other comparison approaches, which suggests the effect of the explicit consideration of using context-fused guidance.

However, the visual relation bias is not well handled. In the future, we will extend our network with scene graph, because it provides a unified representation that connects the objects, attributes, and their relationship in an image or a sentence. It is more advantageous for the model to employ the scene graph to depict an image with an accurate text description about object relationships.

## Figures and Tables

**Figure 1:** The main idea of our proposed network. The compositional visual feature consists of the image representation at regional and global level. At each decoding step, the context gate calculates the textual context by dynamically aggregating the visual concept and word embedding. The context-fused image guidance is formulated on the compositional visual features and fused textual context.

**Figure 2:** The overview of our proposed network. For the visual concept set *A*={*a*_1_, *a*_2_,…, *a*_*m*_}, a unidirectional LSTM is adopted to obtain the encoded vector *w*. The region image feature *r* is extracted by a Faster R-CNN, and the image representation $\bar{r}$ is obtained by the max pooling applied on *r*. In decoder, a two-layer LSTM architecture is adopted. *s*_*t*_ indicates the fused textual context. Both *V*_comp_ and context-fused guidance *g*_*t*_ are passed into the language LSTM along with the hidden state *h*_*t*_^*v*^ from attention LSTM. The input vector *X* consists of $\bar{r}$, *w* the word embedding, and the hidden state of language LSTM.

**Figure 3:** An illustration of the context gate. *f*_*t*_ is the scalar factor, s_t_ is the fused textual context, and *E(y)* indicates the word embedding vectors.

**Figure 4:** Generated captions by the models with different guidance formulation. The positive cases are framed in blue and the failed cases are framed in red.

**Figure 5:** Visualization of the attention map (bottom) and the word probabilities in the generated sentence (histogram) and visual concept set (line). For conciseness, the weights of the visual concept are presented only.

**Table 1:** Statistics of the MS COCO dataset.

Split	Default		Karpathy	
Subset	Image	Caption	Image	Caption
Training	82,783	414,113	113,287	566,738
Validation	40,504	202,654	5000	25,010
Test	40,775	—	5000	25,010

The symbol “—” indicates the data are not public.

**Table 2:** Performance comparisons on MS COCO Karpathy test split under cross-entropy training.

Cross-entropy loss								
Metric	BLEU1	BLEU2	BLEU3	BLEU4	METEOR	ROUGE-L	CIDEr	SPICE
NIC [16]	—	—	—	29.6	—	52.6	94.0	—
SCST [11]	—	—	—	30.0	25.9	53.4	99.4	—
Up-down [4]	77.2	—	—	36.2	27.0	56.4	113.5	20.3
RFNet [17]	76.4	60.4	46.6	35.8	27.4	56.8	112.5	20.5
HAN [20]	77.2	61.2	47.7	36.2	27.5	56.6	114.8	20.6
RAtt-Soft [29]	**79.2**	**61.8**	47.6	**36.9**	**28.3**	**60.9**	114.3	**20.8**
CFG	77.1	61.5	**47.9**	36.8	27.7	56.7	114.0	**20.8**

The best results (%) are highlighted in boldface. The symbol “—” indicates the results are not reported.

**Table 3:** Performance comparisons on MS COCO Karpathy test split under CIDEr-D score optimization.

Sequence-level optimization								
Metric	BLEU1	BLEU2	BLEU3	BLEU4	METEOR	ROUGE-L	CIDEr	SPICE
NIC [16]	—	—	—	31.9	—	54.3	106.3	—
SCST [11]	—	—	—	34.2	26.7	55.7	114.0	—
Up-down [4]	79.8	—	—	36.3	27.7	56.9	120.1	21.4
RFNet [17]	79.1	63.1	48.4	36.5	27.7	57.3	121.9	21.2
HAN [20]	**80.9**	64.6	49.8	37.6	27.8	58.1	121.7	21.5
RAtt-soft [29]	80.4	63.4	48.9	37.5	**28.5**	**61.6**	122.1	**22.1**
CFG	80.5	**64.7**	**50.2**	**38.3**	28.2	58.3	**125.4**	21.6

The best results (%) are highlighted in boldface. The symbol “—” indicates the results are not reported.

**Table 4:** Performance comparison of the ablative models.

Model	Cross-entropy training			CIDEr optimization		
Metric	BLEU4	CIDEr	SPICE	BLEU4	CIDEr	SPICE
CFG_*V*_	36.1	112.8	20.3	37.7	123.9	21.0
CFG_*E*_	36.1	112.9	20.5	37.8	124.6	21.1
CFG_*A*_	36.3	113.0	20.6	38.1	124.6	21.4
CFG	**36.8**	**114.0**	**20.8**	**38.3**	**125.4**	**21.6**

## Data Availability

The data used to support the findings of this study are included within the article.

## References

[1] Chen S., Jin Q., Wang P., Wu Q. Say as you wish: fine-grained control of image caption generation with abstract scene graphs.

[2] Wang H., Zhang Y., Yu X. (2020). An overview of image caption generation methods. *Computational Intelligence and Neuroscience*.

[3] Xu K., Ba J., Kiros R. Show, attend and tell: neural image caption generation with visual attention.

[4] Anderson P., He X., Buehler C. Bottom-up and top-down attention for image captioning and visual question answering.

[5] Huang L., Wang W., Chen J., Wei X.-Y. Attention on attention for image captioning.

[6] Jia X., Gavves E., Fernando B., Tuytelaars T. Guiding long-short term memory for image caption generation.

[7] Zhou L., Xu C., Koch P., Corso J. J. Watch what you just said: image captioning with text-conditional attention.

[8] Jiang W., Ma L., Chen X., Zhang H., Liu W. Learning to guide decoding for image captioning.

[9] Fang H., Gupta S., Iandola F. N., Srivastava R. K., Deng L. From captions to visual concepts and back.

[10] Ranzato M., Chopra S., Auli M., Zaremba W. Sequence level training with recurrent neural networks.

[11] Rennie S. J., Marcheret E., Mroueh Y., Ross J., Goel V. Self-critical sequence training for image captioning.

[12] Vedantam R., Lawrence, Zitnick C., Parikh D. CIDEr: Consensus-based image description evaluation.

[13] Luo R., Shakhnarovich G., Cohen S., Price B. Discriminability objective for training descriptive captions.

[14] Zha Z.-J., Liu D., Zhang H., Zhang Y., Wu F. (2020). Context-aware visual policy network for fine-grained image captioning. *IEEE Transactions on Pattern Analysis and Machine Intelligence*.

[15] Bujimalla S., Subedar M., Tickoo O. (2020). B-SCST: bayesian self-critical sequence training for image captioning. https://arxiv.org/abs/2004.02435.

[16] Vinyals O., Toshev A., Bengio S., Erhan D. Show and tell: a neural image caption generator.

[17] Jiang W., Ma L., Jiang Y.-G., Liu W., Zhang T. Recurrent fusion network for image captioning.

[18] Zheng K., Zhu C., Lu S., Liu Y. Multiple-level feature-based network for image captioning.

[19] Sammani F., Melas-Kyriazi L. Show, edit and tell: a framework for editing image captions.

[20] Wang W., Chen Z., Hu H. Hierarchical attention network for image captioning.

[21] Papineni K., Roukos S., Ward T., Zhu W. J. Bleu: a method for automatic evaluation of machine translation.

[22] Ren S., He K., Girshick R., Sun J. (2017). Faster R-CNN: towards real-time object detection with region proposal networks. *IEEE Transactions on Pattern Analysis and Machine Intelligence*.

[23] Tu Z., Liu Y., Lu Z., Liu X., Li H. (2017). Context gates for neural machine translation. *Transactions of the Association for Computational Linguistics*.

[24] Lin T.-Y., Maire M., Belongie S. Microsoft COCO: common objects in context.

[25] Banerjee S., Lavie A. METEOR: an automatic metric for MT evaluation with improved correlation with human judgments.

[26] Lin C. Y. Rouge: a package for automatic evaluation of summaries.

[27] Anderson P., Fernando B., Johnson M., Gould S. Spice: semantic propositional image caption evaluation.

[28] Kingma D. P., Ba J. (2014). Adam: a method for stochastic optimization. https://arxiv.org/abs/1412.6980.

[29] Zhang Z., Wu Q., Wang Y. (2021). Exploring region relationships implicitly: image captioning with visual relationship attention. *Image and Vision Computing*.

[30] Yang X., Tang K., Zhang H., Cai J. Auto-encoding scene graphs for image captioning.

